The article "Solid lipid curcumin particles provide greater anti-amyloid, anti-inflammatory and neuroprotective effects than curcumin in the 5xFAD mouse model of Alzheimer’s disease" was retracted in 2023. Reasons: errors in the images; duplicated images.

# Solid lipid curcumin particles provide greater anti-amyloid, anti-inflammatory and neuroprotective effects than curcumin in the 5xFAD mouse model of Alzheimer’s disease

**DOI:** 10.1186/s12868-018-0406-3

**Published:** 2018-02-23

**Authors:** Panchanan Maiti, Leela Paladugu, Gary L. Dunbar

**Affiliations:** 1 Field Neurosciences Institute Laboratory for Restorative Neurology, Central Michigan University, Mt. Pleasant, MI 48859 USA; 2 Program in Neuroscience, Central Michigan University, Mt. Pleasant, MI 48859 USA; 3 Department of Psychology, Central Michigan University, Mt. Pleasant, MI 48859 USA; 4 Field Neurosciences Institute, St. Mary’s of Michigan, Saginaw, MI 48604 USA; 5 Department of Biology and Brain Research Laboratory, Saginaw Valley State University, Saginaw, MI 48604 USA

**Keywords:** Alzheimer’s disease, Neurodegeneration, Neuroinflammation, Curcumin, Amyloid beta protein, Anti-amyloid

## Abstract

**Background:**

Neuroinflammation and the presence of amyloid beta protein (Aβ) and neurofibrillary tangles are key pathologies in Alzheimer’s disease (AD). As a potent anti-amyloid and anti-inflammatory natural polyphenol, curcumin (Cur) could be potential therapies for AD. Unfortunately, poor solubility, instability in physiological fluids, and low bioavailability limit its clinical utility. Recently, different lipid modifications in the formulae of Cur have been developed that would enhance its therapeutic potential. For example, we have reported greater permeability and neuroprotection with solid lipid curcumin particles (SLCP) than with natural Cur in an in vitro model of AD. In the present study, we compared the Aβ aggregation inhibition, anti-amyloid, anti-inflammatory responses of Cur and or SLCP in both in vitro and in vivo models of AD. One-year-old 5xFAD-and age-matched wild-type mice were given intraperitoneal injections of Cur or SLCP (50 mg/kg body weight) for 2- or 5-days. Levels of Aβ aggregation, including oligomers and fibril formation, were assessed by dot blot assay, while Aβ plaque load and neuronal morphology in the pre-frontal cortex (PFC) and hippocampus were assayed by immunolabeling with Aβ-specific antibody and cresyl violet staining, respectively. In addition, neuroinflammation was assessed the immunoreactivity (IR) of activated astrocytes (GFAP) and microglia (Iba-1) in different brain areas. Finally, comparisons of solubility and permeability of Cur and SLCP were made in cultured N2a cells and in primary hippocampal neurons derived from E16 pups of 5xFAD mice.

**Results:**

We observed that relative to Cur, SLCP was more permeable, labeled Aβ plaques more effectively, and produced a larger decrease in Aβ plaque loads in PFC and dentate gyrus (DG) of hippocampus. Similarly, relative to Cur, SLCP produced a larger decrease of pyknotic, or tangle-like, neurons in PFC, CA1, and CA3 areas of hippocampus after 5 days of treatment. Both Cur and or SLCP significantly reduced GFAP-IR and Iba-1-IR in PFC, in the striatum as well as CA1, CA3, DG, subicular complex of hippocampus, and the entorhinal cortex in the 5xFAD mice after 5 days of treatment.

**Conclusions:**

The use of SLCP provides more anti-amyloid, anti-inflammatory, and neuroprotective outcomes than does Cur in the 5xFAD mouse model of AD.

**Electronic supplementary material:**

The online version of this article (10.1186/s12868-018-0406-3) contains supplementary material, which is available to authorized users.

## Background

Alzheimer’s disease (AD) is one of the most common, age-related neurodegenerative disorders, affecting millions of people world-wide. It is characterized by selective and progressive neuronal loss, dysfunction of synaptic integrity, and perturbation of neuronal communication, which ultimately leads to memory loss and other cognitive impairments [1]. Aggregation of misfolded amyloid beta protein (Aβ) plaques and hyper-phosphorylated tau (p-tau) are main pathologies [2] and causative factors for producing neuroinflammation and neurodegeneration in AD [3–5]. Although the mechanistic details of Aβ-induced neuroinflammation are not yet clear, it is considered to be one of the primary events which initiate neurodegeneration in AD [4–6]. The neuroinflammation in AD brain involves an activation of microglia and astrocytes around the Aβ plaques [7, 8], which triggers several cascade pathways, including secretion of pro-inflammatory cytokines, such as interleukins (ILs), tumor necrosis factor-α (TNF-α), prostaglandin, nitric oxide (NO), which are all highly associated with neurodegeneration in AD [9–11]. Several studies have been conducted to determine ways to inhibit neuroinflammation in AD. For example, administration of non-steroidal anti-inflammatory drugs (NSAIDs) significantly suppresses the neuroinflammation and improves cognitive and behavioral outcomes in animal models of AD [12], providing a strong rationale for anti-inflammatory therapies for AD pathology.

Several anti-inflammatory drugs have been tested for decreasing neuroinflammation and neurodegeneration in AD. Recently, a potent anti-amyloid natural polyphenol, curcumin (Cur), has become one of the most promising compounds for inhibiting misfolded Aβ aggregation and reducing neuroinflammation [13–15]. It is a bright, yellow-colored pigment, derived from the root of the herb, *Curcuma longa* [16]. Because of its pleiotropic actions, such as anti-amyloid [14, 17], anti-oxidant [18], and anti-inflammatory properties [19], Cur has been targeted for therapeutic applications in AD [15, 20, 21]. Many studies have been performed with Cur to reduce neuroinflammation in both animal models of AD [13, 22–24], and in human patients with AD [25, 26]. Recently, Liu and colleagues [10] found that Cur reduced neuroinflammation in a rat model of AD by activating peroxisome proliferator activator receptor gamma (PPAR-γ). However, the poor solubility, instability in physiological fluids, and low bioavailability of Cur are the major obstacles for effectively delivering it in therapeutically significant amounts [27, 28]. This explains why most of the studies have been performed with chronic administration of Cur to achieve its therapeutic value. However, because of its hydrophobic and lipophilic nature, several investigators have tried to use lipidated formula of Cur, including the use of solid lipid Cur particles (SLCPs), to achieve its greater and faster effects on AD [29]. Recently, we and others have shown that SLCP increases Cur solubility, stability, and bioavailability, and enhances anti-amyloid and anti-inflammatory activities, while providing neuroprotection in both pre-clinical and clinical trials design to test its efficacy for treating AD [15, 20, 24, 26, 30, 31].

Given this, the present study was designed to compare the effects of acute treatments of Cur and or SLCP on anti-inflammatory activities, Aβ plaque loads, and neuronal morphology in different brain regions of 5xFAD mice. Our results suggest that the SLCP permeated brain tissue, reduced neuroinflammation and lessened Aβ plaque loads in 5xFAD mice more effectively than did Cur.

## Methods

### Chemicals

Curcumin (Cur, ~ 65% pure), Aβ42, 1,1,1,3,3,3-Hexafluoro isopropanol (HFIP) and other accessory chemicals were procured from Sigma (St. Louis, MO). The glial fibrillary acidic protein (GFAP) and Iba-1 (ionized calcium-binding adapter molecule 1) antibodies were purchased from Abcam (Cambridge, MA) and Wako (Richmond, VA), respectively. The Aβ oligomer specific (A11) and fibril specific antibodies (OC) were purchased from Chemicon International (Billerica, Massachusetts), and 6E10 was purchased from BioLegend (San Diego, CA). Solid lipid curcumin particles (SLCP, which contains 26% Cur) was gifted from the Verdure Sciences (Noblesville, IN). This SLCP consists of high-purity, long-chain phospholipid bilayer and a long-chain fatty acid solid lipid core, which coats the Cur. The SLCP has been well characterized by us [32] and others in vitro, animal models [30, 33–35] and in clinical trials of AD [26].

### Animals

Thirty-two, one-year-old B6SJL-Tg (APPSwFlLon, PSEN1*M146L*L286V, 1136799Vas/J; Jackson Laboratory, stock no: 34840-JAX/5xFAD) and age-matched wild-type mice (N = 4 in each group) were used in this study. The 5xFAD mice overexpressed human APP and PS1 with five familial AD mutations, including three mutations on APP gene [Swedish (K670N, M671L), Florida (I716V), and London (V717I)] and two on PS1 gene (M146L and L286V) [36, 37]. A detailed pathology of these mice was described previously [32, 38–40]. All mice were housed at 22 °C under a 12-h light/12-h dark, reverse-light cycle with *ad libitum* access of food and water. All mice were genotyped at 3 weeks of age by polymerase chain reaction (PCR) to confirm their transgenic characteristics, as reported previously [41]. This study was carried out in strict accordance with the protocols approved by the Institutional Animal Care and Use Committee of the Central Michigan University (IACUC 09-13A). All surgeries were performed under isoflurane anesthesia, and all efforts were made to minimize animal discomfort.

#### Injection of Cur or SLCP to 5xFAD mice

Age-matched wild-type and 5xFAD mice (1-year-old) were injected intraperitoneally (i.p.) with Cur or SLCP for 2 and 5 days. The mice were randomly divided into eight groups (n = 4 each group): Group-I (wild type; WT); Group-II (WT + Cur-5 days); Group-III (WT + SLCP-5 days); Group-IV (5xFAD); Group-V (5xFAD + Cur-2 days); Group-VI (5xFAD + Cur-5 days); Group-VII (5xFAD + SLCP-2 days) and Group-VIII (5xFAD + SLCP-5 days). The Cur and SLCP were dissolved in methanol and diluted in 0.1 M PBS (pH 7.4, final methanol concentration was < 1%) and injected (i.p., at 50 mg/kg) one a day to mice in groups: II, III, V, VI, VII and VIII. The same volume of vehicle (PBS) was injected to WT (Group I) and 5xFAD mice (Group-IV), as summarized in Table 1.

**Table 1:** Summary of the different animal groups and treatment regimens used in this study

Groups	Mouse genotype	Treatments	Number of mice used/group	Duration of treatment (days)
I	WT	PBS	4	5
II	WT	Cur	4	5
III	WT	SLCP	4	5
IV	5xFAD	PBS	4	5
V	5xFAD	Cur	4	2
VI	5xFAD	Cur	4	5
VII	5xFAD	SLCP	4	2
VIII	5xFAD	SLCP	4	5

#### Tissue processing

All mice were deeply anaesthetized with an overdose of sodium pentobarbital (i.p.), and transcardially perfused with 0.1 M cold PBS at pH 7.4, followed by 4% paraformaldehyde (diluted in 0.1 M PBS at pH 7.4) to fix the brains. The brains were then removed, suspended in 4% paraformaldehyde for 24 h at 4 °C, and transferred to the graded sucrose solutions (10, 20 and 30%). When brains were completely immersed in the 30% sucrose solution, they were stored at 4 °C until being sectioned coronally at 40 µm on a Cryostat (Leica, Germany).

#### Cur and SLCP permeability study

To investigate whether sufficient amounts of Cur or SLCP crossed the blood brain barrier (BBB) and reached to the regions of interest in the brain, the Cur- and the SLCP-injected 5xFAD mice (Group V–VIII) were sacrificed and their brain tissue was processed, as described above. Coronal sections (40 μM) were cut and imaged using a fluorescent microscope (Leica, Germany) to assess the amount of Cur or SLCP bound to the Aβ plaques, which was confirmed by co-localization of either the Cur or the SLCP to Aβ-specific antibody (6E10) in Aβ-plaques, as described previously [32]. To compare the permeability of Cur and SLCP in vitro, mouse neuroblastoma cells (N2a, ATCC, Catalog no: Neuro2a (ATCC^®^ CCL131™) and the primary hippocampal neurons from a 5xFAD mouse were used. The N2a cells were grown with minimum essential medium (MEM, GIBCO) containing 10% heat-inactivated fetal bovine serum (FBS), and penicillin and streptomycin (100 I.U./mL and 100 μg/mL). The culture was maintained at 37 °C in a humidified atmosphere at 5% CO_2_. The primary hippocampal neurons were taken from embryonic-16 (E16) mouse pups and grown in neurobasal media containing B27 supplementation for 7 days in vitro (7-DIV), as described previously [42]. Prior to the experiment, the cells were grown in either in 60 mm Petri dishes or on glass coverslips, using fresh MEM or neurobasal media that lacked growth factors. The cells were then treated with 100 μM of either Cur or SLCP for 2 h, after which the media was removed, and the cells were fixed with 4% paraformaldehyde solution. Microphotographic images were taken using a fluorescent microscope (Leica, Germany) with appropriate excitation/emission filters for analyses.

#### Aβ plaque load in 5xFAD after treatment with Cur or SLCP

To check the effects of acute treatment of Cur or SLCP on Aβ plaque burden, the 5xFAD brain sections were stained with Cur and the number of Aβ plaques were counted in these sections. Cur was used to label Aβ plaques, because it labels plaques as efficiently as Aβ-specific antibody [32]. Using Image-J software (http://imagej.nih.gov/ij), the total area of each image was measured and the numbers of Aβ plaques were counted manually in PFC and DG area of hippocampus and expressed as number of Aβ plaques per 100 µm^2^ area. Only clearly visible, large fluorescent signals were considered as Aβ plaques. A minimum of 10 serial sections, with forty different fields were used to count the number of Aβ plaques in each group (n = 4), with the experimenters blinded to the group identity of the specimens analyzed.

#### Neuronal morphology by cresyl violet staining

One of the aims of this study was to investigate whether short-term treatment of Cur or SLCP can protect the neuronal morphology, especially in hippocampal subfields and in the PFC area. To this end, the tissue from 5xFAD mice that were treated with Cur or SLCP was stained with 0.1% cresyl violet, as described previously [43]. The sections were washed, dehydrated, cleared, mounted, and coverslipped using DePex mounting media (BDH, Batavia, IL). The slides were dried, after which photomicrographs were taken using a compound light microscope (Olympus, Japan) with 100× objectives (total magnification of 1000×). The number of pyknotic, or tangle-like, cells were counted manually using Image-J software (http://imagej.nih.gov/ij), and were expressed as number of pyknotic cells per 100 µm^2^ area. A minimum of 5 serial sections, each with 10 different fields, were used for counting the number of pyknotic cells in each group (n = 4), with the experimenters blinded to the group identity of the specimens being analyzed.

#### Neuroinflammation study by immunohistochemistry

To compare the anti-inflammatory effects of Cur or SLCP in 5xFAD mice, the brain tissue from each mouse was labeled with GFAP and Iba-1, which are the markers for activated astrocytes and microglia, respectively.

##### GFAP-immunohistochemistry

A subset of brain sections were rinsed three times with 0.1 M PBS (pH 7.4) for 5 min each. The sections were then blocked with 10% normal goat serum for 1 h at room temperature with gentle shaking. The tissue was incubated overnight on a shaker at 4 °C with GFAP antibody (rabbit polyclonal, 1:500). On the next day, the sections were thoroughly washed with PBS, three times, for 10 min each. The sections were incubated with anti-rabbit secondary antibody (1:1000), tagged with Alexa-594 (Molecular Probes, OR), for 30 min at room temperature. Then sections were washed thoroughly with distilled water, dehydrated, cleared and mounted on slides using anti-fading Fluoro-mount aqueous mounting media (Sigma) prior to microscopic examination using a fluorescence microscope (Leica, Germany) with the appropriate excitation/emission filters.

##### Iba-1 immunohistochemistry

Similarly, for Iba-1 immunohistochemistry, another subset of brain section were thoroughly rinsed, three times with 0.1 M PBS (pH 7.4) for 5 min each. The sections were then immersed in a solution of 3% hydrogen peroxide and 0.1 M PBS (pH 7.4) for 30 min at room temperature to inhibit endogenous peroxidase. Then the sections were rinsed with PBS and blocked with 10% normal goat serum (NGS), which underwent gently shaking for 1 h at room temperature. The tissue was then incubated with Iba-1 antibody (rabbit, monoclonal, 1:4000) with gentle shaking for 4 h at room temperature and then for overnight at 4 °C. On the next day, the sections were thoroughly washed 3 times for 5 min each, and incubated with biotinylated anti-rabbit secondary antibody (1:250) for 1 h at room temperature. Finally, the sections were incubated with peroxidase substrate solution, supplied with the ABC kit (Vector Laboratory, CA), and the signal was developed using diaminobenzidine (DAB) until the desired staining intensity emerged. The tissue was then washed, dehydrated with graded alcohol, cleared with xylene, mounted on slides, coverslipped with DePex (BDH, Batavia, IL), air dried, and visualized using a compound light microscope (Olympus, Japan) with 20× objectives (total magnification 200×).

#### Quantification of GFAP-IR and Iba-1-IR cells

For quantification of GFAP-IR and Iba-1-IR cells, the sections were imaged using a fluorescent microscope (Leica, Germany) and a compound light microscope (Olympus, Japan), respectively. The number of GFAP-IR and Iba-1-IR were counted manually using Image-J software (http://imagej.nih.gov/ij). Briefly, the images were taken from randomly selected regions of the layer IV/V of PFC (bregma +3.20 mm), striatum (bregma +1.00 mm), subicular complex, hippocampus (CA1, CA3 and dentate gyrus) at bregma −3.30 mm, and the entorhinal cortex (bregma −3.30 mm), using 20× objectives (total magnification at 200×). The total area of each image was measured and the numbers of GFAP-IR and Iba-1-IR cells were counted manually in those areas. Only clearly visible fluorescent signals or brown DAB color were considered as GFAP-IR and Iba-1-IR cells, respectively. The GFAP-IR and Iba-1-IR cells were expressed as number of cells per 100 µm^2^ area. A minimum of 10 serial sections, from which thirty different fields were used to count the number of GFAP-IR and Iba-1-IR cells in each group, using four different animals in each group with the experimenter blinded to the group identity of the specimens analyzed.

#### Comparative study of inhibition of Aβ42 aggregation by Cur or SLCP

To compare the anti-amyloid activity, such as inhibition of Aβ42 oligomer and fibril formation by Cur or SLCP, the dot blot assay was used [14]. Briefly, Aβ42 peptide was dissolved in HFIP, vortexed for 1 min and allowed to solubilize for 30 min at room temperature. Then, the HFIP was evaporated under laminar hood, until the peptide was completely dried to make a thin film. This was followed by speed-vacuuming for 10 min [42, 44], after which the film was stored at − 20 °C. Each HFIP film was dissolved in 60 mM NaOH (final concentration 6 mM) and diluted with Tris-buffer saline (TBS, 0.1 M, pH 7.4, 0.025% NaN3) to get the desired peptide concentration (10 μM). Then 50 μL of peptide solution (10 μM) was taken in Eppendorf tube and incubated, with or without different concentrations of Cur or SLCP (in μM: 1, 0.1, 0.01, 0.001), for 8-, and 24-h at 37 °C, with gentle shaking (200 rpm). After the stipulated period of incubation, about 10 μL of peptide solution was spotted on nitrocellulose membrane (Bio-Rad, CA, USA). Then, the membrane was blocked with 5% nonfat milk in TBS-Tween-20 (TBS-T) at room temperature for 1 h, washed with TBS-T, and probed with Aβ-oligomer (A11) and Aβ fibril (OC) specific antibodies (rabbit polyclonal, 1: 1000) in 5% non-fat milk powder in TBS-T overnight at 4 °C. After washing, it was probed with anti-rabbit horseradish-peroxidase (HRP) conjugated secondary antibody solution (1: 25,000, Santa Cruz Biotech, CA, USA) for 1 h at room temperature. After washing three times, the blot was developed with Amersham ECL Prime Western Blot Detection Reagent (GE-Healthcare Life Sciences, PA, USA) for 2–5 min. The dot blots were scanned using gel documentation system (Bio-Rad, CA, USA), and the optical density of each dot was measured using Image-J software (http://imagej.nih.gov/ij).

### Statistical analysis

The morphometric data for GFAP-IR and Iba-1-IR in different brain areas were expressed as mean ± SEM. All data were analyzed using one way analysis of variance (ANOVA) with Tukey HSD (honest significant difference) *post*-*hoc* tests being conducted when appropriate. A probability value ≤ 0.05 was considered as statistically significant.

## Results

### Comparison of permeability of Cur or SLCP to the brain tissue

To compare the permeability of Cur or SLCP after their injections (i.p.) for 2 or 5 days, the 5xFAD mouse brains were sectioned and observed under a fluorescent microscope. We observed that both Cur and SLCP crossed the BBB and bound with Aβ plaques after 2- and 5-days of injections (Fig. 1a) and co-localized with Aβ-specific antibody (6E10) (Fig. 1b). We also found that SLCP showed more permeability than Cur, as assessed by intensity of fluorescent signals that were bound with Aβ plaques. In addition, those mice receiving 5 days of treatment showed increased Aβ plaque labeling when compared to those receiving 2 days of treatment for both the Cur and SLCP groups (Fig. 1a). Similarly, a trend towards more solubility and greater permeability was observed after 2 h exposure of SLCP over Cur with N2a and primary hippocampal neurons at 7 days in vitro (Additional file 1: Fig. S1).

**Fig. 1:** Curcumin or SLCP cross the blood brain barrier and binds with amyloid plaques. After intraperitoneal injections of Cur or SLCP (50 mg/kg), the 5xFAD brains were sectioned and images were taken from DG area of hippocampus using a fluorescent microscope with green filters. **a** Both Cur and SLCP permeated into the brain tissue, and SLCP appeared to be more permeable than Cur, and those receiving 5 days of treatment appeared to have more Cur in the brain than those receiving only 2 days of injections. **b** Images of sections from the DG area of the hippocampus in the Cur- or SLCP-treated mice were immunolabeled with Aβ-specific antibody (6E10) as observed by using a fluorescent microscope with green and red filters. Cur or SLCP colocalized with 6E10, confirming the green signal coming from Aβ plaques upon binding with Cur or SLCP. Red arrows: Cur or SLCP bound to the Aβ plaque; green arrow: 6E10 bound to Aβ plaque; and white arrow: merged images of Cur or SLCP and 6E10 with Aβ plaque. Scale bars indicate 250 µm and is applicable to other images

### Cur or SLCP treatment decreased Aβ plaque load in 5xFAD mice brain

After stipulated periods of Cur or SLCP treatment in 5xFAD mice, the brain sections were stained with SLCP (100 µM) (Fig. 2a) and Aβ-specific antibody (6E10) (Fig. 2b), followed by counts of the number of Aβ plaques. We observed that after 5 days of treatment with Cur or SLCP, the number of Aβ plaques were significantly decreased (*p* < 0.01) in the PFC (Cur: 49% and SLCP: 56.31%) (Fig. 2c) and in DG area of hippocampus (Cur: 36.30% and SLCP: 50.50%) (Fig. 2d) in comparison to vehicle-treated 5xFAD group. Further, SLCP-treated mice had fewer Aβ plaques than did Cur-treated mice (Fig. 2c, d). Similarly, our dot blot assays showed that both Cur and SLCP significantly inhibited Aβ42-oligomers (Fig. 3a–c) and fibril formation (Fig. 3d–f). However, SLCP treatment showed significantly greater inhibition (*p* < 0.01) of Aβ42 fibril formation after 24 h of treatment than did Cur (Fig. 3d–f).

**Fig. 2:** Acute treatment of either Cur or SLCP reduced Aβ plaque loads in 5xFAD mice brain. **a** The 5xFAD mice were treated with Cur or SLCP for 2- or 5-days, sacrificed, and their brains were sectioned on a cryostat and stained with Cur, which labeled the Aβ plaques that were observed in the PFC and the DG area of the hippocampus. Scale bar indicates 250 µm and is applicable to the other images. **b** Cur binds to Aβ plaques in a manner similar to Aβ-specific antibody (6E10), so it was used for labeling and counting Aβ plaques in this study. Scale bar indicates 100 µm and is applicable to the other images. **c**, **d** The number of Aβ plaques were significantly decreased (**p < 0.01) in both the PFC (**c**) and the DG area of the hippocampus (**d**) in comparison to untreated 5xFAD mice

**Fig. 3:** SLCP inhibits Aβ fibril formation greater than does Cur. Aβ42 peptide was dissolved in HFIP, and after being completely dried, it was dissolved in 60 mM NaOH and diluted with Tris buffer saline (1 mM, pH 7.4), yielding a 10 μM concentration. Fifty microliter of peptide solution was incubated with, or without, different concentrations of Cur or SLCP for 8- and 24-h. After the stipulated period for each experiment, about 10 μL of peptide solution was spotted on the nitrocellulose membrane. The blots were probed with Aβ-oligomer specific (A11) and fibril specific (OC) antibodies. **a**–**c** inhibition of Aβ42-oligomer formation by Cur and SLCP.** d**–**f** Aβ42 fibril formation was attenuated by Cur and SLCP after 24 h of incubation. Note that SLCP showed greater inhibition of Aβ42 fibril formation than dietary Cur (**d**,** e**). Results were expressed as mean ± SEM from three independent experiments. **p < 0.01 and ***p < 0.001 in comparison to Aβ42-vehicle treated group

### Neuronal morphology in the 5xFAD mouse brain after treatment with Cur or SLCP

One of the aims of this study was to investigate whether short-term treatment of Cur or SLCP can protect neuronal morphology. Therefore, the treated brain tissue was stained with cresyl violet and many pyknotic or tangle-like neuron, along with vacuolization within the pyramidal cell layers, were observed in PFC, CA1, and CA3 subfields of hippocampus in the 5xFAD mice. After 5 days of Cur or SLCP treatment (but not at 2 days of treatment), we observed significant decreases (*p* < 0.01) of pyknotic, or tangled-like, cells in PFC (Cur: 27%; SLCP: 33%; Fig. 4a, b), in CA1 (Cur: 24%; SLCP: 36%; Fig. 4a, c) and in CA3 area (Cur: 13%; SLCP: 26%; Fig. 4a, d) of the hippocampus.

**Fig. 4:** Cur and SLCP treatments partially protect neuronal morphology in the 5xFAD mice brain tissue. The 5xFAD mice were treated with Cur or SLCP for 2- or 5-days, sacrificed, and the subsequent cryostat sections were stained with 0.1% cresyl violet, from which images were taken using Olympus microscope (total magnification: 1000x) in the PFC and the CA1 and CA3 regions of hippocampus. **a** Pyknotic, tangle-like, neurons along with vacuoles were observed in 5xFAD tissue with Cur- or SLCP-treatment reducing this abnormal morphology in the PFC and hippocampal neurons following 5-, but not 2-days of treatment. **b** The number of pyknotic cells were less after 5 days of treatment (*p < 0.05; **p < 0.01) in all three areas, when compared to the 5xFAD mice receiving only vehicle or the 5xFAD mice receiving only 2 days treatment. Scale bar indicates 25 µm and is applicable to other images. Arrows indicate pyknotic or tangle-like neurons

### Changes in microglial morphology after treatment with Cur or SLCP in 5xFAD mice

To investigate the changes of microglial morphology after treatment with Cur or SLCP, the 5xFAD brain sections were immunolabeled with Iba-1 antibody. There was profound branching and intense expression of Iba-1 protein in 5xFAD tissue, whereas treatment with Cur or SLCP appeared to decrease the number of branches and the amount of Iba-1 levels in PFC and in different subfields of hippocampus, as well as in the striatum after both 2- and 5-days of treatment with Cur or SLCP (Fig. 5). We also observed that the levels of Iba-1 and the extent of microglial branching tended to be less only in the 5-days treatment group in comparison to the 2-day group.

**Fig. 5:** Morphological changes of single microglial cells in the 5xFAD mouse brain after treatment with Cur or SLCP. The 5xFAD mice were treated with Cur or SLCP for 2- or 5-days, sacrificed, and their brain sections were immunolabeled for Iba-1 antibody. The Iba-1-IR appeared to be more intense and the branching of microglia were more diffuse in the brain tissue of the vehicle-treated 5xFAD mice compared to those mice treated with Cur or SLCP for either 2- or 5-days. Scale bar indicates 250 µm and is applicable to all images

### Microglial aggregation morphology after treatment with Cur or SLCP in 5xFAD mice

When we looked at the morphology of microglial aggregation, or clumping, we observed that there was a noticeable aggregation of microglia in the vehicle-treated 5xFAD group, which was less noticeable in the brain tissue of mice treated with Cur or SLCP, with the latter groups also showing a reduction in Iba-1 labeling (Fig. 6). Further, we found a trend towards less aggregation of microglia and Iba-1-IR in 5xFAD mice given 5 days of Cur or SLCP treatment, relative to those receiving 2 days of treatment and with those given SLCP showing less microglial aggregation in comparison to those given Cur (Fig. 6).

**Fig. 6:** Morphological changes of aggregated microglia in 5xFAD mice brains after treatment with Cur or SLCP. The 5xFAD mice were treated with Cur or SLCP for 2- or 5-days, sacrificed, and their brain sections were immunolabeled for Iba-1 antibody. The tissue from the vehicle-treated 5xFAD mice showed significant clumping, or aggregation of activated microglia, whereas, those of 5xFAD mice that were treated with Cur or SLCP for 2- or 5-days had fewer aggregations of microglia and less intense labeling of Iba-1. Scale bar indicates 250 µm and is applicable to all images

### Morphological changes of astrocytes after treatment with Cur or SLCP in 5xFAD mice

Similar to the microglial changes, we have also investigated the morphological changes of activated astrocytes by immunolabeling with GFAP antibodies after treatment with Cur or SLCP in 5xFAD mice. The brains of the 5xFAD mice showed activation of astrocytes, as evidenced by extensive branching, along with increased level of GFAP-IR, whereas brains of the 5xFAD treated with Cur or SLCP appeared to have decreased activation, with a trend toward less GFAP-IR and astrocyte branching in the PFC and in different subfields of the hippocampus (Fig. 7). We did not find any significant differences in morphology of activated astrocytes between the 5xFAD mice given Cur or SLCP, whether the treatments were given for 2- or 5-days.

**Fig. 7:** Morphological changes of activated astrocytes from brain tissue of 5xFAD mice after treatment with Cur or SLCP. The 5xFAD mice were treated with Cur or SLCP for 2- or 5-days, sacrificed, and the subsequent cryostat sections were immunolabeled with GFAP antibody. The GFAP immunofluorescence appeared to be more intense and the branching of astrocytes was more extensive in vehicle-treated 5xFAD mice, compared with those given Cur or SLCP for 2- or 5-days. Scale bar indicates 250 µm and is applicable to other images

### Cur and SLCP treatments decreased Iba-1-IR and GFAP-IR in PFC of 5xFAD mice

When we counted the number of Iba-1-IR cells in PFC, we observed that Cur or SLCP treatments significantly decreased (*p* < 0.01) the number of Iba-1-IR cells in comparison to those of the untreated 5xFAD mice (Fig. 8a, b). In addition, 5 days of either SLCP or Cur treatment showed greater reduction (*p* < 0.05) of Iba-1-IR in comparison to 2 days of treatment. Furthermore, SLCP showed greater reduction of Iba-1-IR in comparison to those given Cur for either 2- or 5-days (Fig. 8a, b). Similar findings were observed for counts of GFAP-IR cells in the PFC (Fig. 8a, c).

**Fig. 8:** Cur or SLCP treatment reduces neuroinflammation in the PFC of 5xFAD mice. The 5xFAD mice were treated with either Cur or SLCP for 2- or 5-days, sacrificed, and their brain sections were collected and immunolabeled for Iba-1 and GFAP. The number of Iba-1-IR- (**a**, **b**) and GFAP-IR- (**a**, **c**) labeled cells was significantly reduced (*p < 0.05; **p < 0.01) in the PFC in all Cur- and SLCP-treated mice in comparison to untreated 5xFAD mice. Further reduction was observed after 5-, relative to 2-, days of treatment, for both the GFAP and Iba-1 labeling (**b**, **c**). Scale bar indicates 250 µm and is applicable to other images

### Cur and SLCP treatments decreased Iba-1-IR and GFAP-IR in CA1 region of hippocampus of 5xFAD mice

One of our interests was to investigate the neuroinflammation profile in hippocampal subfields of 5xFAD mice after acute treatment with Cur or SLCP. We observed that both Cur and or SLCP significantly decreased (*p* < 0.01) Iba-1-IR and GFAP-IR cells in CA1 region, in comparison to vehicle-treated 5xFAD mice (Fig. 9a–c). We also found a significant difference (*p* < 0.05) between the 2- and 5-day treatment groups in Iba-1-IR labeling and between the Cur and SLCP groups (*p* < 0.05) (Fig. 9b), but these differences were not observed for GFAP labeling (Fig. 8a, c).

**Fig. 9:** Cur and SLCP treatments reduce neuroinflammation in CA1 subfield of hippocampus in 5xFAD mice. The 5xFAD mice were treated with Cur or SLCP for 2- or 5-days, sacrificed, and their brain sections were collected and immunolabeled for Iba-1 and GFAP. The number of labeled Iba-1-IR (**a**,** b**) and GFAP-IR (**a**,** c**) cells were significantly reduced (*p < 0.05; **p < 0.01) in the CA1 area, in comparison to vehicle-treated 5xFAD mice, with further reductions were observed after 5 days of treatment, compared with that of at 2 days (**b, c**). Scale bar indicates 250 µm and is applicable to other images

### Cur and SLCP treatments decreased Iba-1-IR and GFAP-IR in CA3 region of hippocampus of 5xFAD mice

Similar to CA1 region, there was a significant decrease (*p* < 0.01) in the number of Iba-1-IR and GFAP-IR in CA3 subfield of hippocampus after treatment with either Cur or SLCP (Fig. 10a–c). The Iba-1-IR was less in the 5-day SLCP group, relative to the 2-day SLCP group (*p* < 0.01) (Fig. 10b). No differences of GFAP-IR were observed between 2- and 5-day treatment groups were observed, irrespective of whether the 5xFAD mice received Cur or SLCP (Fig. 10a, c).

**Fig. 10:** Cur and SLCP treatments reduce neuroinflammation in CA3 region of hippocampus in 5xFAD mice. The 5xFAD mice were treated with Cur or SLCP for 2- and 5-days, sacrificed, and their brain sections were collected and immunolabeled for Iba-1 and GFAP. The number of Iba-1-IR (**a**, **b**) and GFAP-IR (**a**, **c**) labeled cells were significantly reduced (*p < 0.05; **p < 0.01) in the CA3 region of hippocampus in comparison to untreated 5xFAD mice. Further reduction was observed after 5 days, in comparison to 2 days, of treatment in the amount of labeling for both GFAP and Iba-1 (**b**, **c**). Scale bar indicates 250 µm and is applicable to other images

### Cur and SLCP treatments decreased Iba-1-IR and GFAP-IR in dentate gyrus of hippocampus of 5xFAD mice

The number of Iba-1-IR and GFAP-IR cells were significantly less (*p* < 0.01) in DG area in Cur- and or SLCP-treated mice, as was the case with the CA1 and CA3 regions (Fig. 11a–c). There were significant decreases in Iba-1-IR between the 2- and 5-day groups given treatment of either of Cur (*p* < 0.01) or SLCP (*p* < 0.01) (Fig. 11b). In addition, the SLCP treatment reduced Iba-1-IR at both 2-and and 5-day treatment periods, relative to what was observed with Cur (Fig. 11b). Similarly, there were significant decreases (*p* < 0.05) in GFAP-IR after 5 days, relative to 2 days, following either Cur or SLCP treatment (Fig. 11a, c). Differences in GFAP-IR measures were also observed between Cur and SLCP treatments (*p* < 0.05) at 2 days, but not at 5 days of treatment (Fig. 11a, c).

**Fig. 11:** Cur and SLCP treatments reduce neuroinflammation in DG area of hippocampus in 5xFAD mice. The 5xFAD mice were treated with Cur or SLCP for 2- or 5-days, sacrificed, and their brain sections were collected and immunolabeled for Iba-1 and GFAP. The number of Iba-1-IR (**a**,** b**) and GFAP-IR (**a**,** c**) were significantly reduced (*p < 0.05; **p < 0.01) in the DG area of hippocampus in comparison to untreated 5xFAD mice. Further reduction was observed after 5-, relative to 2-, days of treatment in the amount for both GFAP and Iba-1 labeling (**b**, **c**). Scale bar indicates 250 µm and is applicable to other images

### Cur and SLCP treatments decreased Iba-1-IR and GFAP-IR in subicular complex of 5xFAD mice

The subicular complex lies between the entorhinal cortex and the CA1 subfield of the hippocampus proper and is very important for neurotransmission from the hippocampus to the cortex. We found a significant decrease (*p* < 0.01) in Iba-1-IR cells in subicular complex in the 5 versus the 2-day, groups treated with Cur (Fig. 12a, b). In addition, SLCP treatment decreased Iba-1-IR in both the 2- and 5-day treatment groups, in comparison to Cur (Fig. 12a, b). Similar findings were also observed in the case of GFAP-IR in these regions (Fig. 12a, c).

**Fig. 12:** Cur and SLCP treatments reduce neuroinflammation in subicular complex of hippocampus in 5xFAD mice. The 5xFAD mice were treated with Cur or SLCP for 2- or 5-days, sacrificed, and their brain sections were collected and immunolabeled for Iba-1 and GFAP. The number of Iba-1-IR (**a**, **b**) and GFAP-IR (**a**, **c**) cells were significantly reduced (*p < 0.05; **p < 0.01) in subicular complex of hippocampus of Cur- or SLCP-treated, versus vehicle-treated 5xFAD mice. Further reduction was observed after 5 days of treatment in comparison to 2 days, of treatment for both GFAP and Iba-1 labeling in both the Cur- and SLCP-treated 5xFAD mice (**b**, **c**). Scale bar indicates 250 µm and is applicable to other images

### Cur and SLCP treatments decreased Iba-1-IR and GFAP-IR in entorhinal cortex of 5xFAD mice

The entorhinal cortex is the major input and output structure of the hippocampal formation and is involved in the maintenance of cortico-hippocampal circuits. The number of Iba-1-IR microglia were significantly decreased (*p* < 0.01) in both the 2- and 5-day Cur or SLCP treatment groups (Fig. 13a, b). Significant decreases (*p* < 0.01) of Iba-1-IR cells were observed in the 5-day group in comparison to 2-day group, with the SLCP-treated mice having fewer Iba-1-IR cells than those receiving Cur (Fig. 13a, b). In contrast, 2 days Cur treatment did not reduce the number of GFAP-IR astrocytes, whereas both Cur and SLCP significantly decreased (*p* < 0.01) GFAP-IR after 5 days of treatment. We also found there was a significant decrease (*p* < 0.01) in the GFAP-IR between the Cur and SLCP groups after 5 days of treatment (Fig. 13a, c).

**Fig. 13:** Cur and SLCP reduce neuroinflammation in entorhinal cortex in 5xFAD mice. The 5xFAD mice were treated with Cur or SLCP for 2- or 5-days, sacrificed, and their brain sections were collected and immunolabeled for Iba-1 and GFAP. The number of labeled Iba-1-IR (**a**, **b**) and GFAP-IR (**a**, **c**) cells was significantly reduced (**p < 0.01) in the entorhinal cortex in comparison to vehicle-treated 5xFAD mice. Significant reduction in both GFAP-IR and Iba-1-IR was observed after 5 days, in comparison to those receiving 2 days, of treatment (**b**, **c**). Scale bar indicates 250 µm and is applicable to other images

### Cur and SLCP treatments decreased Iba-1-IR and GFAP-IR in striatum of 5xFAD mice

The striatum is a subcortical part of the forebrain and is a critical component of the reward system, as well as playing a role in learning and memory. Similar to the other brain structures, the striatum had fewer (*p* < 0.01) Iba-1-IR and GFAP-IR cells than in control mice after 2- and 5-day of either Cur or SLCP treatment (Fig. 14a–c), with the SLCP treatments providing greater reductions than Cur on both of these parameters (Fig. 14a–c).

**Fig. 14:** Cur or SLCP reduce neuroinflammation in the striatum of 5xFAD mice. The 5xFAD mice were treated with Cur or SLCP for 2- and 5-days, sacrificed, and their brain sections were collected and immunolabeled for Iba-1 and GFAP. The number of Iba-1-IR (**a**, **b**) and GFAP-IR (**a**, **c**) labeled cells was significantly reduced (**p < 0.01) in the striatum in comparison to untreated 5xFAD mice. Significant reductions were observed after 5 days, in comparison to 2 days of treatment, on measures of both GFAP and Iba-1 labeling (**b**, **c**). Scale bar indicates 250 µm and is applicable to other images

## Discussion

Because of its unique physicochemical, anti-amyloid, and anti-inflammatory properties, Cur is being considered as a potential treatment for AD [13, 15, 45, 46]. The objectives of the present study were to: (1) compare the permeability of Cur and SLCP into the brain; (2) compare anti-inflammatory activities of Cur with those of SLCP after acute treatment in 5xFAD mice; (3) assess microglial and astrocytic activation in different brain regions, especially those areas associated with AD, after treatment with Cur and or SLCP; and (4) determine which short-term treatment protocol (2 or 5 days) with Cur or SLCP would most effectively decrease Aβ plaque loads and reduce aberrant neuronal morphology in different brain parts of 5xFAD mice. We found that, following short-term i.p. injections, both Cur or SLCP permeated into the brain in therapeutically significant amounts, decreased Aβ plaque loads, and improved neuronal morphology after 5 days of treatment. Both Cur and SLCP also decreased the GFAP-IR and Iba-1-IR in different brain areas of 5xFAD mice. The SLCP tended to confer more effective anti-amyloid, anti-inflammatory, and neuroprotective effect, than did Cur.

Unfortunately, the low solubility in body fluids and its rapid degradation after intestinal absorption limit the bioavailability of natural Cur, reducing its clinical utility for treating AD [15, 28]. However, the use of SLCP, a lipidated formula of Cur, shows significant promise in providing greater neuroprotective effects in animal models [31, 32] and clinical trials of AD [26]. In the present study, we observed that SLCP tended to have greater affinity to Aβ plaques, compared to Cur. Our findings suggest that the lipid bilayer of SLCP facilitates its permeability into the brain. Further, we observed that after 5 days of intraperitoneal injection of either Cur or SLCP, an increase in binding to Aβ plaque was observed, indicating that more Cur accumulates in the tissue with extended treatment. Although we did not measure the free Cur concentration in the brain tissues of the Cur- or SLCP-treated mice, we have previously found 300–400 nM of free Cur in the mouse brain and 2–3 folds more in their plasma, when mice were fed orally for 2 months [24, 30–32, 47] with a similar formula of Cur, when given at a dose of 500 ppm. This was also observed during a clinical trial of AD [26]. Moreover, we have compared the permeability of Cur in different cells, such as 7-DIV primary hippocampal neurons and N2a cells (Additional file 1: Fig. S1) and found that SLCP tended to deliver more free Cur into the cells than did natural Cur [31, 32]. In addition, we also compared the Aβ-binding capability of Cur and or SLCP, in the brain tissue of 5xFAD mice given i.p. injections of Cur or SLSP, observed significant amounts of Cur and SLCP reached the brain and that SLCP appeared to provide greater binding to Aβ plaques in comparison to Cur. We hypothesize that SLCP may have greater capability of delivering free Cur in the brain tissue than Cur (Fig. 1) [32]. However, further investigations with different Cur formulae are needed to confirm and extend these findings in order to optimize this form of therapy.

When we compared the number of Aβ plaques in prefrontal cortex (PFC) and dentate gyrus (DG) of the hippocampus in both Cur- and SLCP-treated 5xFAD mice, we found that after 5-, but not 2-days, of treatment, a significant reduction (~ 50%) of Aβ plaques in PFC and DG areas was observed in both the Cur and SLCP groups (Fig. 2), suggesting the longer duration of treatment is required to optimize reduction in plaque load. Interestingly, after 5 days of treatment, the size or the plaques was relatively smaller and breakage or disaggregation of plaques by Cur or SLCP was confirmed [14, 17]. We have carefully counted the number of Aβ plaques on single focal plane, but more work using unbiased stereology is needed to confirm those findings and provide a more comprehensive profile of the effects of these treatments on Aβ plaques. Nonetheless, we observed greater reductions of Aβ plaques in case of SLCP group, which may be due to its higher permeability into brain tissue, when compared to that of Cur, allowing it to become more capable of inhibiting the assembly of Aβ plaques (Fig. 2). In our dot blot experiments, SLCP also appeared to inhibit Aβ fibril formation more than that observed by Cur, which may be due higher penetration of free Cur released by the SLCPs, which interspersed between Aβ species and interfered with their aggregation pathway (Fig. 3). Although we have yet to directly measure the levels of soluble Aβ after treatment with Cur and or SLCP in 5xFAD mice, we have shown that SLCP reduced Aβ-oligomer formation more than did Cur, as shown by our dot blot experiment (Fig. 3). Similarly, we have shown the number of Aβ plaques were significantly reduced in the PFC and hippocampus (Fig. 2), which indicates that Cur and SLCP can reduce soluble Aβ, as reported by several researchers previously [14, 48, 49].

One of the aims of the present study was to investigate whether short-term treatments of Cur or SLCP could provide neuroprotection. To this end, we have investigated neuronal morphology using cresyl-violet stained tissue. Interestingly, we observed a significant decrease (30%) in the number of pyknotic, or tangle-like, neurons in PFC, CA1, and CA3 subfields of hippocampus after 5 days of either Cur- or SLCP-treatment, but not after 2 days (Fig. 4). This finding suggests that increasing the duration of Cur- or SLCP-treatments may be required to achieve optimal neuroprotection. Although the exact mechanism of neuroprotection following Cur-treatment remains to be delineated, several investigators have demonstrated that Cur can stimulate numerous neurotropic factors, including increases in brain derived neurotropic factor (BDNF), glial derived neurotropic factor (GDNF), and nerve growth factor (NGF), which preserve the function and viability of neurons [10, 50, 51]. Increased in trophic factors may underlie the reduction in pyknotic cells in the SLCP-treated 5xFAD mice, relative to those receiving Cur, and this which may be due to the presence of more Cur in the brain made available due to the greater permeability of SLCP.

As a potent anti-inflammatory polyphenol, Cur can also produce its therapeutic effects by reducing neuroinflammation in AD via activation of cytokine production, as well as the inhibition of the NF-kB signaling pathway [10]. We found that Cur and SLCP treatments significantly reduced microglial activation (Iba-1-IR) in different brain regions. Surprisingly, when we investigated the morphology of microglial aggregation, we observed a significant reduction of both microglia arborization and the level of Iba-1-IR, which suggests that both Cur and SLCP may inhibit activation of microglia (Fig. 6), as reported by others [10]. Similarly, both Cur and SLCP treatments significantly decreased GFAP-IR and branching of astrocytes by inhibiting their activation (Fig. 7). When we counted the number of GFAP-IR and Iba-1-IR cells in different brain areas, especially, in the PFC, CA1, CA3, DG, subiculum, entorhinal cortex, and striatum, we observed an inhibition of Iba-1-IR and GFAP-IR in the Cur- and or SLCP-treated mice. The GFAP-IR and Iba-1-IR profile in hippocampal subfields and the areas associated with hippocampus, especially subicular complex and entorhinal cortex, the junctional areas which connect with cortex, revealed that 5 days of either Cur- or SLCP-treatment reduced neuroinflammation to a greater extent than 2 days of treatment, which, again, suggests that a longer duration of treatment is required to optimize the anti-inflammatory effects of Cur and or SLCP. Interestingly, we achieved greater anti-inflammatory effects in the case of SLCP treatment, which, again, confirmed that the SLCP facilitates permeability of Cur across the blood brain barrier (BBB) so it can inhibit neuroinflammation to a greater degree than Cur. Although we did not investigate the molecular mechanism of inhibition of reactive microglia and astrocytes after Cur or SLCP treatments, others [10] have demonstrated that Cur attenuates Aβ-induced neuroinflammation by activating the peroxisome proliferator-activated receptor-gamma (PPAR-γ) in a rat model of AD. Indeed, Cur can reduce neuroinflammation by inhibiting the NF-kB [52] and ERK [53] signaling pathways, which are regulated by PPAR-γ [10]. Moreover, Cur also inhibits other inflammatory cytokines, by inhibiting further activation of astrocytes and microglia in AD brain [14, 54, 55].

## Conclusions

As a potent, anti-amyloid and anti-inflammatory natural polyphenol, Cur is a promising therapy for AD. It significantly reduced neuroinflammation as measured by GFAP and Iba-1 immunoreactivity in different key brain areas of 5xFAD mice after acute treatment. Short-term treatment of Cur and or SLCP decreased amyloid plaque load and reduced abnormal neuronal morphology in 5xFAD mice. The SLCP treatments provided greater anti-inflammatory, anti-amyloid and neuroprotective effects compared to Cur in 5xFAD mice. Taken together, our data suggest that SLCP reduces neuropathology to a greater extent in animal models of AD than does Cur, and, therefore, may provide a more efficient and effective treatment for AD.

## Additional file

**Additional file 1: Fig. S1.** Comparative solubility and permeability of Cur or SLCP in vitro. A: schematic diagram of formulation of SLCP. Upper row: Solubility of Cur and SLCP in PBS. Note SLCP appeared to be more soluble in PBS, whereas Cur predominantly formed crystal-like structures. Middle and lower rows: The SLCP appeared to confer greater permeability than Cur in both N2a and 7-DIV primary hippocampal neurons after 2 h of incubation.

## Abbreviations

AD: Alzheimer’s disease
Cur: curcumin
SLCP: solid lipid curcumin particles
5xFAD: 5x-familial Alzheimer’s disease
GFAP: glial fibrillary acidic protein
Iba-1: ionized calcium-binding adapter molecule
IR: immunoreactivity
Aβ: amyloid beta protein
IL: interleukin
TNF-α: tumor necrosis factor-α
NO: nitric oxide
PBS: phosphate buffer saline
NSAIDs: non-steroidal anti-inflammatory drugs
PPAR-γ: peroxisome proliferator-activated receptor gamma
APP: amyloid precursor protein
PSEN1: presenilin-1
PCR: polymerase chain reaction
PFC: prefrontal cortex
DG: dentate gyrus
ABC: avidin biotin complex
DAB: diaminobenzidine
ANOVA: analysis of variance
HSD: honest significant difference
CV: cresyl violet
BDNF: brain derived neurotropic factor
GDNF: glial derived neurotropic factor
NGF: nerve growth factor
NF-kβ: nuclear factor kappa beta
ERK: extracellular signal-regulated kinase
AU: arbitrary unit
DIV: day in vitro

## References

[1] Campbell VA, Gowran A (2007). Alzheimer’s disease; taking the edge off with cannabinoids?. Br J Pharmacol.

[2] Selkoe DJ (2004). Cell biology of protein misfolding: the examples of Alzheimer’s and Parkinson’s diseases. Nat Cell Biol.

[3] Szekely CA, Thorne JE, Zandi PP, Ek M, Messias E, Breitner JC, Goodman SN (2004). Nonsteroidal anti-inflammatory drugs for the prevention of Alzheimer’s disease: a systematic review. Neuroepidemiology.

[4] Zhang F, Jiang L (2015). Neuroinflammation in Alzheimer’s disease. Neuropsychiatr Dis Treatm.

[5] Bronzuoli MR, Iacomino A, Steardo L, Scuderi C (2016). Targeting neuroinflammation in Alzheimer’s disease. J Inflamm Res.

[6] Parajuli B, Sonobe Y, Horiuchi H, Takeuchi H, Mizuno T, Suzumura A (2013). Oligomeric amyloid beta induces IL-1beta processing via production of ROS: implication in Alzheimer’s disease. Cell Death Dis.

[7] Mandrekar-Colucci S, Landreth GE (2010). Microglia and inflammation in Alzheimer’s disease. CNS Neurol Disord: Drug Targets.

[8] Cameron B, Landreth GE (2010). Inflammation, microglia, and Alzheimer’s disease. Neurobiol Dis.

[9] Akiyama H, Barger S, Barnum S, Bradt B, Bauer J, Cole GM, Cooper NR, Eikelenboom P, Emmerling M, Fiebich BL (2000). Inflammation and Alzheimer’s disease. Neurobiol Aging.

[10] Liu ZJ, Li ZH, Liu L, Tang WX, Wang Y, Dong MR, Xiao C (2016). Curcumin attenuates beta-amyloid-induced neuroinflammation via activation of peroxisome proliferator-activated receptor-gamma function in a rat model of Alzheimer’s disease. Front Pharmacol.

[11] Kitazawa M, Yamasaki TR, LaFerla FM (2004). Microglia as a potential bridge between the amyloid beta-peptide and tau. Ann N Y Acad Sci.

[12] McGeer PL, McGeer EG (2007). NSAIDs and Alzheimer disease: epidemiological, animal model and clinical studies. Neurobiol Aging.

[13] Lim GP, Chu T, Yang F, Beech W, Frautschy SA, Cole GM (2001). The curry spice curcumin reduces oxidative damage and amyloid pathology in an Alzheimer transgenic mouse. J Neurosci.

[14] Yang F, Lim GP, Begum AN, Ubeda OJ, Simmons MR, Ambegaokar SS, Chen PP, Kayed R, Glabe CG, Frautschy SA (2005). Curcumin inhibits formation of amyloid beta oligomers and fibrils, binds plaques, and reduces amyloid in vivo. J Biol Chem.

[15] Hu S, Maiti P, Ma Q, Zuo X, Jones MR, Cole GM, Frautschy SA (2015). Clinical development of curcumin in neurodegenerative disease. Expert Rev Neurother.

[16] Prasad S, Aggarwal BB, Benzie IFF, Wachtel-Galor S (2011). Turmeric, the golden spice: from traditional medicine to modern medicine. Herbal medicine: biomolecular and clinical aspects.

[17] Ono K, Hasegawa K, Naiki H, Yamada M (2004). Curcumin has potent anti-amyloidogenic effects for Alzheimer’s beta-amyloid fibrils in vitro. J Neurosci Res.

[18] Menon VP, Sudheer AR (2007). Antioxidant and anti-inflammatory properties of curcumin. Adv Exp Med Biol.

[19] Ray B, Lahiri DK (2009). Neuroinflammation in Alzheimer’s disease: different molecular targets and potential therapeutic agents including curcumin. Curr Opin Pharmacol.

[20] Frautschy SA, Cole GM (2010). Why pleiotropic interventions are needed for Alzheimer’s disease. Mol Neurobiol.

[21] McClure R, Yanagisawa D, Stec D, Abdollahian D, Koktysh D, Xhillari D, Jaeger R, Stanwood G, Chekmenev E, Tooyama I (2015). Inhalable curcumin: offering the potential for translation to imaging and treatment of Alzheimer’s disease. J Alzheimer’s Dis JAD.

[22] Lu Z, Cui M, Zhao H, Wang T, Shen Y, Dong Q (2014). Tissue kallikrein mediates neurite outgrowth through epidermal growth factor receptor and flotillin-2 pathway in vitro. Cell Signal.

[23] Griffin WS, Sheng JG, Royston MC, Gentleman SM, McKenzie JE, Graham DI, Roberts GW, Mrak RE (1998). Glial-neuronal interactions in Alzheimer’s disease: the potential role of a ‘cytokine cycle’ in disease progression. Brain Pathol.

[24] Begum AN, Jones MR, Lim GP, Morihara T, Kim P, Heath DD, Rock CL, Pruitt MA, Yang F, Hudspeth B (2008). Curcumin structure-function, bioavailability, and efficacy in models of neuroinflammation and Alzheimer’s disease. J Pharmacol Exp Ther.

[25] Baum L, Lam CW, Cheung SK, Kwok T, Lui V, Tsoh J, Lam L, Leung V, Hui E, Ng C (2008). Six-month randomized, placebo-controlled, double-blind, pilot clinical trial of curcumin in patients with Alzheimer disease. J Clin Psychopharmacol.

[26] Koronyo Y, Biggs D, Barron E, Boyer DS, Pearlman JA, Au WJ, Kile SJ, Blanco A, Fuchs DT, Ashfaq A (2017). Retinal amyloid pathology and proof-of-concept imaging trial in Alzheimer’s disease. JCI Insight.

[27] Anand P, Kunnumakkara AB, Newman RA, Aggarwal BB (2007). Bioavailability of curcumin: problems and promises. Mol Pharm.

[28] Kumar A, Ahuja A, Ali J, Baboota S (2010). Conundrum and therapeutic potential of curcumin in drug delivery. Crit Rev Ther Drug Carrier Syst.

[29] Ghalandarlaki N, Alizadeh AM, Ashkani-Esfahani S (2014). Nanotechnology-applied curcumin for different diseases therapy. Biomed Res Int.

[30] Ma QL, Zuo X, Yang F, Ubeda OJ, Gant DJ, Alaverdyan M, Teng E, Hu S, Chen PP, Maiti P (2013). Curcumin suppresses soluble tau dimers and corrects molecular chaperone, synaptic, and behavioral deficits in aged human tau transgenic mice. J Biol Chem.

[31] Maiti P, Dunbar GL (2017). Comparative neuroprotective effects of dietary curcumin and solid lipid curcumin particles in cultured mouse neuroblastoma cells after exposure to Abeta42. Int J Alzheimer’s Dis.

[32] Maiti P, Hall TC, Paladugu L, Kolli N, Learman C, Rossignol J, Dunbar GL (2016). A comparative study of dietary curcumin, nanocurcumin, and other classical amyloid-binding dyes for labeling and imaging of amyloid plaques in brain tissue of 5x-familial Alzheimer’s disease mice. Histochem Cell Biol.

[33] DiSilvestro RA, Joseph E, Zhao S, Bomser J (2012). Diverse effects of a low dose supplement of lipidated curcumin in healthy middle aged people. Nutr J.

[34] Nahar PP, Slitt AL, Seeram NP (2015). Anti-inflammatory effects of novel standardized solid lipid curcumin formulations. J Med Food.

[35] Cox KH, Pipingas A, Scholey AB (2015). Investigation of the effects of solid lipid curcumin on cognition and mood in a healthy older population. J Psychopharmacol.

[36] Xu F, Kotarba AE, Ou-Yang MH, Fu Z, Davis J, Smith SO, Van Nostrand WE (2014). Early-onset formation of parenchymal plaque amyloid abrogates cerebral microvascular amyloid accumulation in transgenic mice. J Biol Chem.

[37] Maya-Vetencourt JF, Carucci NM, Capsoni S, Cattaneo A (2014). Amyloid plaque-independent deficit of early postnatal visual cortical plasticity in the 5XFAD transgenic model of Alzheimer’s disease. J Alzheimer’s Dis JAD.

[38] Oakley H, Cole SL, Logan S, Maus E, Shao P, Craft J, Guillozet-Bongaarts A, Ohno M, Disterhoft J, Van Eldik L (2006). Intraneuronal beta-amyloid aggregates, neurodegeneration, and neuron loss in transgenic mice with five familial Alzheimer’s disease mutations: potential factors in amyloid plaque formation. J Neurosci.

[39] Kimura R, Ohno M (2009). Impairments in remote memory stabilization precede hippocampal synaptic and cognitive failures in 5XFAD Alzheimer mouse model. Neurobiol Dis.

[40] Ohno M, Chang L, Tseng W, Oakley H, Citron M, Klein WL, Vassar R, Disterhoft JF (2006). Temporal memory deficits in Alzheimer’s mouse models: rescue by genetic deletion of BACE1. Eur J Neurosci.

[41] Sadleir KR, Eimer WA, Cole SL, Vassar R (2015). Abeta reduction in BACE1 heterozygous null 5XFAD mice is associated with transgenic APP level. Mol Neurodegener.

[42] Maiti P, Lomakin A, Benedek GB, Bitan G (2010). Despite its role in assembly, methionine 35 is not necessary for amyloid beta-protein toxicity. J Neurochem.

[43] Maiti P, Singh SB, Muthuraju S, Veleri S, Ilavazhagan G (2007). Hypobaric hypoxia damages the hippocampal pyramidal neurons in the rat brain. Brain Res.

[44] Bitan G, Kirkitadze MD, Lomakin A, Vollers SS, Benedek GB, Teplow DB (2003). Amyloid beta -protein (Abeta) assembly: Abeta 40 and Abeta 42 oligomerize through distinct pathways. Proc Natl Acad Sci USA.

[45] Garcia-Alloza M, Borrelli LA, Rozkalne A, Hyman BT, Bacskai BJ (2007). Curcumin labels amyloid pathology in vivo, disrupts existing plaques, and partially restores distorted neurites in an Alzheimer mouse model. J Neurochem.

[46] Koronyo-Hamaoui M, Koronyo Y, Ljubimov AV, Miller CA, Ko MK, Black KL, Schwartz M, Farkas DL (2011). Identification of amyloid plaques in retinas from Alzheimer’s patients and noninvasive in vivo optical imaging of retinal plaques in a mouse model. Neuroimage.

[47] Hickey MA, Zhu C, Medvedeva V, Lerner RP, Patassini S, Franich NR, Maiti P, Frautschy SA, Zeitlin S, Levine MS (2012). Improvement of neuropathology and transcriptional deficits in CAG 140 knock-in mice supports a beneficial effect of dietary curcumin in Huntington’s disease. Mol Neurodegener.

[48] Shytle RD, Tan J, Bickford PC, Rezai-Zadeh K, Hou L, Zeng J, Sanberg PR, Sanberg CD, Alberte RS, Fink RC (2012). Optimized turmeric extract reduces beta-Amyloid and phosphorylated Tau protein burden in Alzheimer’s transgenic mice. Curr Alzheimer Res.

[49] Thapa A, Jett SD, Chi EY (2016). Curcumin attenuates amyloid-beta aggregate toxicity and modulates amyloid-beta aggregation pathway. ACS Chem Neurosci.

[50] Liu ZJ, Liu W, Liu L, Xiao C, Wang Y, Jiao JS (2013). Curcumin protects neuron against cerebral ischemia-induced inflammation through improving PPAR-gamma function. Evid Based Complement Altern Medicine eCAM.

[51] Lu Z, Shen Y, Wang T, Cui M, Wang Z, Zhao H, Dong Q (2014). Curcumin promotes neurite outgrowth via reggie-1/flotillin-2 in cortical neurons. Neurosci Lett.

[52] Becaria A, Bondy SC, Campbell A (2003). Aluminum and copper interact in the promotion of oxidative but not inflammatory events: implications for Alzheimer’s disease. J Alzheimer’s Dis JAD.

[53] Giri RK, Rajagopal V, Kalra VK (2004). Curcumin, the active constituent of turmeric, inhibits amyloid peptide-induced cytochemokine gene expression and CCR5-mediated chemotaxis of THP-1 monocytes by modulating early growth response-1 transcription factor. J Neurochem.

[54] Mishra S, Palanivelu K (2008). The effect of curcumin (turmeric) on Alzheimer’s disease: an overview. Ann Indian Acad Neurol.

[55] Gupta SC, Prasad S, Kim JH, Patchva S, Webb LJ, Priyadarsini IK, Aggarwal BB (2011). Multitargeting by curcumin as revealed by molecular interaction studies. Nat Prod Rep.

